The article "Protective effect of MiR-146 on renal injury following cardiopulmonary bypass in rats through mediating NF-κB signaling pathway" was retracted in 2024. Reasons: original data or images not available; unreliable results or conclusions; concerns about the data; concerns about the results or conclusions.

# Protective effect of MiR-146 on renal injury following cardiopulmonary bypass in rats through mediating NF-κB signaling pathway

**DOI:** 10.1080/21655979.2021.2012405

**Published:** 2021-12-29

**Authors:** Hongbo Ma, Yanjiao Dong, Kun Sun, Shuo Wang, Zheng Zhang

**Affiliations:** Department of Nephrology, Zibo Central Hospital, Zibo, PR China

**Keywords:** MiR-146, NF KB signaling pathway, rat, cardiopulmonary bypass, renal injury, protective effect

## Abstract

The mechanism of renal injury after cardiopulmonary bypass is not clear, and the protective effect of microRNA-146 through mediating NF KB signaling pathway needs to be verified. The study intends to establish a rat model of cardiopulmonary bypass (CPB). MiR-146 is silenced or overexpressed by lentivirus transfection. It is divided into miR-146 inhibitors group (inhibitors), miR-146 mimics group (mimics) and sham group. It is found that the contents of Cr, bun and MDA in blood = , serum IL-1, IL-6 and TNF in mimics group are higher than those in the other two groups- α Content, apoptosis rate, ICAM-1, TNF- α, NF- κ B mRNA and NF- κ B protein decreased significantly (P < 0.05), while the content of SOD in kidney increased significantly (P < 0.05). In the inhibitors group, the above indicators showed the opposite results. Double luciferase assay showed that NF-kB was the target gene of miR-146. It can be seen that the expression of miR-146 inhibits inflammatory factors, apoptosis, oxidative stress and NF- κ the activation of B pathway promotes the repair of renal injury in CPB rats.

## Introduction

The microcirculatory perfusion is impaired during and after cardiopulmonary bypass (CPB), that is, the CPB decreases the microcirculatory perfusion and increases the heterogeneity of microcirculatory perfusion distribution, which may lead to tissue oxygenation derangement, thus resulting in tissue injury [1,2]. The microcirculatory perfusion injury is an inverse predictor of the prognosis of critically ill patients, and it is considered to play a vital role in the development of organ dysfunction [3,4]. Experimental studies have manifested that the CPB can reduce the perfused vessel density, enhance the activation of endothelial cells and impair the renal oxygenation [5,6]. In addition, the increased hematocrit during the CPB ameliorates the microcirculatory perfusion of the patients in the Department of Cardiac Surgery [7]. The CPB is also the second most common cause of acute kidney injury (AKI) in the ICU, so it is particularly worthy of study as the time of renal injury is predictable and the mechanism of the disease is relatively uniform [8]. With the decline in glomerular filtration rate, conventional markers of renal injury, including serum creatinine (Cr), are accumulated in the blood, but they are still the golden standard for renal injury. Even the mild AKI can increase the morbidity and mortality rates of the hospitalized patients, especially the critically ill patients [9]. Therefore, studies on multiple intervention measures for preventing or treating AKI have been conducted, some of which have obtained preferable data from animal models, while the results of clinical trials are usually disappointing [10]. Delayed diagnosis and uncertain pathogenesis of human AKI may make some explanation on these failures. Despite the considerable time and efforts invested by researchers, there is still a lack of successful intervention measures for the treatment of related diseases to renal injury. Hence, it is urgent to seek for new therapeutic methods to provide bases for the prevention and treatment of renal injury and its complications.

The article "Protective effect of MiR-146 on renal injury following cardiopulmonary bypass in rats through mediating NF-κB signaling pathway" was retracted in 2024. Reasons: original data or images not available; unreliable results or conclusions; concerns about the data; concerns about the results or conclusions.

The functions of micro ribonucleic acids (miRNAs) in the pathogenesis of diversified diseases has been fully explored in studies, and miRNAs play vital roles in physiology and various diseases [11]. As non-coding RNAs, miRNAs participate in protein coding and specific regulation of non-coding genes, and increasingly more investigations have demonstrated that a third of the human genes are probably regulated by miRNAs [12]. Besides, miRNAs can be involved in the regulation of multiple processes such as cell cycle, metabolism and diversified immune responses [13], and they have become crucial regulatory factors of gene expression in many diseases, whose regulatory networks have been paid much attention to in recent years [14]. According to a study, miR-146 is down-regulated in the early stage of hepatic ischemia/reperfusion (I/R) injury, and miR-146a can participate in the regulation of arthritis mainly by negatively regulating the immuno-inflammatory responses, thereby exerting important effects in cell proliferation [15]. Nuclear factor-kappa B (NF-κB) transcription factor are ubiquitous and capable of controlling numerous biological processes such as inflammation and cell apoptosis [16]. NF-κBp65 is the most common in cells, and p65 is the key player in the cell apoptosis triggered by tumor necrosis factor-alpha (TNF-α) and can significantly inhibit TNF-α to protect organisms from the damage of TNF-α-induced toxicity [17]. Therefore, the dysregulated NF-κB will become a pathogenic impetus. However, the potential role of miR-146 in renal injury and the action mechanism in modulating NF-κB in rats have not been clarified yet, which need to be verified by more studies. Hence, the present study proposed that miR-146 can protect against renal injury in the CPB rats through the NF-κB signaling pathway.

The article "Protective effect of MiR-146 on renal injury following cardiopulmonary bypass in rats through mediating NF-κB signaling pathway" was retracted in 2024. Reasons: original data or images not available; unreliable results or conclusions; concerns about the data; concerns about the results or conclusions.

This study aims to investigate the influence of miR-146 on renal injury in the CPB rats through the NF-κB signaling pathway, which was elaborated by the establishment of the CPB model, overexpression and silencing of miR-146, in-vivo experiments and multiple molecular biological techniques. Finally, the specific molecular mechanism of action of such influence was explored. In a word, the experimental results in this study enrich and improve the theoretical bases for the influences of miR-146 on the CPB-associated renal injury and the NF-κB signaling pathway, thereby revealing the protective effect of miR-146 on the CPB-associated renal injury.

## 1. Materials and methods

### 1.1 Reagents and instruments

Enzyme-linked immunosorbent assay (ELISA) kits for interleukin-1 (IL-1), IL-6, superoxide dismutase (SOD), etc. (Nanjing SenBeiJia Biological Technology Co., Ltd.), RIPA lysis buffer (Beyotime Institute of Biotechnology), SDS-PAGE loading buffer, protease inhibitor and bicinchoninic acid (BCA) protein assay kit (Biosharp), β-actin and secondary antibodies (Beijing Ray Antibody Biotech), primary antibodies (Cell Signaling Technology), tissue homogenizer (HaimenAiband Laboratory Equipment Co., Ltd.), EPS 300 electrophoresis apparatus (Bio-Rad, USA), Multiskan MK3 microplate reader (Thermo Fisher Scientific, USA), 2500 gel imager (Bio-Rad, USA), quantitative polymerase chain reaction (qPCR) instrument (7900 Fast, Applied Biosystems, USA), TRIzol reagent and DEPC-treated water (Medical Discovery Leader), UltraPure Agarose, SuperScript III reverse transcription (RT) kit and SYBR qPCR Mix (ABI), and pipette (Eppendorf).

### 1.2 Animal modeling and grouping

All the experiments were approved by the Animal Ethics Committee of Tongji Hospital, Tongji Medical College, Huazhong University of Science and Technology. All Sprague-Dawley rats were fed adaptively in conventional cages for a week and had free access to food and water. The right jugular vein was punctured, and the venous blood was drained into a CPB circuit through a bypass pump, oxygenated in a small animal-specific membrane oxygenator and pumped into the caudal artery. The perfusion flow was set at about 40 mL/kg/min at the beginning of bypass, then gradually increased to 100 mL/kg/min, maintained for 1 h and finally decreased stepwise to stop. When the rats resuscitated completely, they were put back into the cages and fasted, with free access to water. The rats in Sham group underwent the same operations except for the CPB. On the basis of CPB, miR-146 was transfected and overexpressed via amplification using gene-specific primers, and the purified and recovered reaction products were ligated with vector fragments under the action of T4 deoxyribonucleic acid (DNA) Ligase, and the ligation products were transformed into competent cells. Later, miR-146 expression was transferred into adenovirus vectors and then transfected into the rats. Subsequently, the rats were divided into miR-146 inhibitors group (Inhibitors group, n = 20) and miR-146 mimics group (Mimics group, n = 20), and the reaction was continued for 24 h for subsequent experiments.

The article "Protective effect of MiR-146 on renal injury following cardiopulmonary bypass in rats through mediating NF-κB signaling pathway" was retracted in 2024. Reasons: original data or images not available; unreliable results or conclusions; concerns about the data; concerns about the results or conclusions.

### 1.3 Transfection of miR-146 in each group of rats

To deeply investigate the protective effect of miR-146 on the CPB-associated renal injury in rats, miR-146 was transfected into the rats by virtue of adenovirus. Later, the transfection efficiency of miR-146 in the kidney was detected via RT-PCR, making preparations for subsequent studies on the molecular mechanism of miR-146 in protecting the CPB-associated renal injury.

### 1.4 Detection of renal function in each group of rats

Abnormal changes in the renal function may occur after the CPB-associated renal injury in rats so, for the purpose of predicting the incidence of renal injury and providing crucial references for early diagnosis in clinical practices, the renal function indexes such as Cr and blood urea nitrogen (BUN) were examined. The blood (4 mL) was collected from the caudal vein under sterile conditions and centrifuged at 3,000 g and low temperature for 10 min. Then the supernatant was harvested and subpackaged in centrifuge tubes. Finally, the changes in the levels of related indexes in the serum were determined using a fully-automatic biochemistry analyzer according to the operating instructions.

### 1.5 Observation of changes in renal tissues via hematoxylin and eosin (HE) staining

After anesthesia with pentobarbital, the rats were sacrificed in a sterile environment, and the renal tissues were isolated, soaked in formalin and then washed with running water for 24 h, followed by clearing, dipping and embedding in paraffin. The paraffin blocks were made into about 5 μm-thick pathological sections, stained with hematoxylin for 15 min, flushed in water and counterstained in eosin for 5 min, followed by dehydration in alcohol, transparentization and sealing with neutral balsam. Finally, the tissues were observed under a light microscope.

### 1.6 Detection of content of inflammatory factors via ELISA

The content of serum inflammatory factors was measured by means ELISA. 4 mL of tail vein blood was drawn aseptically and centrifuged at 3,000 g and low temperature for 10 min to collect the supernatant, which was subpackaged in 200 μL centrifuge tubes. Next, the samples to be detected (100 μL) were incubated at 37°C for 60 min and washed, and the changes in the indexes were detected by kits according to the practical situation and specific instructions. Ultimately, the absorbance of the inflammatory factors in each group was measured using the microplate reader.

The article "Protective effect of MiR-146 on renal injury following cardiopulmonary bypass in rats through mediating NF-κB signaling pathway" was retracted in 2024. Reasons: original data or images not available; unreliable results or conclusions; concerns about the data; concerns about the results or conclusions.

### 1.7 Detection of levels of oxidant and anti-oxidant indexes SOD and malondialdehyde (MDA) in renal tissues via ELISA

After the rats were anesthetized and sacrificed, the renal tissues were harvested and washed with normal saline. Then 0.5 g of renal tissues were broken using the homogenizer containing prepared tissue lysis buffer, followed by centrifugation at 2000 × g for 15 min, acquisition of supernatant and detection of changes in SOD and MDA levels. At last, the absorbance of the indexes in each group was measured using the microplate reader, and the standard curves were plotted to analyze the changes in the content in accordance with the specific instructions.

### 1.8 TUNEL detects renal apoptosis

According to the TUNEL cell apoptosis detection kit (Roche), the prepared paraffin sections were tested for myocardial tissue apoptosis. The sealed section samples were labeled with a fluorescent color reagent, fixed, rinsed, and permeated with 0.1% Triton X-100, and TUNEL positive cells were observed. The FITC-labeled TUNEL-positive cells at 530 nm were excited at 488 nm under a fluorescence microscope, and 10 fields of view were taken to count the TUNEL-positive cells.

### 1.9 Detection of expression of relevant genes via RT-PCR

[1] The rats in each group were anesthetized with pentobarbital and killed under sterile conditions, and the renal tissues were separated. Then, 100 mg of aseptic renal tissue was carefully and accurately weighed at low temperature, ground with the addition of liquid nitrogen, and the lysis buffer was added for homogenization at 2,200 r/min and low temperature for 15 s. The total RNA was extracted from the tissues, and its concentration was ensured qualified [2]. Primer amplification was conducted using a 20 μL system [2 μL of complementary DNA (cDNA), 10 μL of Mix, 2 μL of primer and 6 μL of ddH_2_O] for 40 cycles, and messenger RNA (mRNA) was synthesized into cDNA and then stored for later use [3]. Later, PCR amplification was performed according to pre-denaturation at 95°C for 2 min, and PCR at 94°C for 20 s, 60°C for 20 s and 72°C for 30 s, 40 cycles in total. The sequences of target genes and internal reference [glyceraldehyde-3-phosphate dehydrogenase (GAPDH)] were designed based on those on GenBank(Table 1). The expression levels of target genes were detected via qRT-PCR. The relative expression levels of related genes in each group of renal tissues were calculated using 2^−ΔΔCt^ method.

The article "Protective effect of MiR-146 on renal injury following cardiopulmonary bypass in rats through mediating NF-κB signaling pathway" was retracted in 2024. Reasons: original data or images not available; unreliable results or conclusions; concerns about the data; concerns about the results or conclusions.

**Table 1.** The primer sequence of each index in RT-PCR

target gene	Primer sequence (5′–3′)
GAPDH	F:5ʹ-TGACTTCAACAGCGACACCCA-3 R:5ʹ-CACCCTGTTGCTGTAGCCAAA-3
TNF-α	F:5ʹ- CGCTACGACCGCCAG ATTG-3ʹ R:5ʹ- ACACCGTTCACCAGCAAGTC-3’
ICAM-1	F:5ʹ-CCCGTAAATCGAAGCTAATG-3ʹ R:5ʹ-TTAAGGCATCCAGTCCGAGT-3’
NF-KB MIR-146 SOD	F:5ʹ -CTGAACCAGGGCATACCTGT-3ʹ R:5ʹ- GAGAAGTCCATGTCCGCAAT-3ʹ F:5ʹ-CGTATCCAGTGCAGGGTCCGA-3 R:5ʹ-TTCGCACTGGATACGACCCCC-3 F:5ʹ- TTCAATAAGGAGCAGGGAC-3ʹ R:5ʹ- CAGTGTAAGGCTGACGGTTT-3’

### 1.10 Western blotting assay

[1] The rats were anesthetized by pentobarbital and then killed under sterile conditions, and the renal tissues were isolated, 150 mg of which were precisely weighed and placed in 10 mL Eppendorf (EP) tubes. After grinding at low temperature, the tissues were rapidly broken using the homogenizer at low temperature, followed by centrifugation and collection of the supernatant [2]. Then the supernatant was subpackaged into the EP tubes, and the protein concentration was detected and calculated in accordance with the instructions of BCA kit [3]. The total proteins in the renal tissues were extracted, prepared into samples, subjected to water bath for 8 min and centrifuged at 1,000 g for 5 min. After that, Western blotting assay was performed as follows: The proteins were loaded for electrophoresis, transferred onto membrane and then incubated with primary antibodies and secondary antibodies. The protein bands were scanned and quantified using a membrane scanner (Bio-Rad), the level of proteins to be detected was corrected by GAPDH, and the grayscale value of the protein bands was analyzed through ImageLab.

### 1.11 Dual luciferase reporter experiment

Take the logarithmic growth phase human embryonic kidney HEK293 cells provided by the American ATCC company. LipofetamineTM2000 liposome transfection reagent was used to transfect the wild-type plasmid vector NF-KB-WT and the mutant plasmid vector NF-KB-MUT into HEK293 cells, respectively. At the same time, MIR-146 mimics and MIR-146 inhibitors were separately transfected into HEK293 cells. After 24 hours of transfection, the cells were collected and lysed. The relative luciferase activity was detected with a luciferase kit, and the transcription activity of the target gene was analyzed.

### 1.12 Statistical analysis

The original recorded data of the experiment were processed with SPSS 20.0 analysis software, and the data were multi-compared. The experimental results obtained were expressed as mean ± standard deviation (x± SD), and statistically significant difference was P < 0.05. The histogram uses GraphPad prism 5.0.

The article "Protective effect of MiR-146 on renal injury following cardiopulmonary bypass in rats through mediating NF-κB signaling pathway" was retracted in 2024. Reasons: original data or images not available; unreliable results or conclusions; concerns about the data; concerns about the results or conclusions.

## 2 Results

### 2.1 Transfection results of miR-146 in each group of rats

In this experiment, 40 rats successfully constructed a CPB model. The success rate of CPB-related kidney injury in rats was 100%. The expected experiment, specimen retention, and detection operations were successfully completed. In order to observe the transfection efficiency of miR-146 in each group of rats, the gene expression level was detected. It was indicated that the expression level of miR-146 was elevated extremely notably in Mimics group and lowered markedly in Inhibitors group (*p* < 0.05), suggesting that the transfection efficiency was prominent, and related verification tests could be further conducted (Figure 1).

**Figure 1.** Transfection effect of MIR-146b the expression of MIR-146 in the Mimics group increased, and the content in the inhibitors group decreased (P < 0.05) **P < 0.05.

### 2.2 Serum detection results of renal function

Such vital biochemical indexes as Cr and BUN in the serum have important functions in nephropathy, so their content was measured by the conventional biochemistry analyzer. The results (Table 2) showed that Mimics group exhibited evidently decreased content of Cr and BUN, while Inhibitors group manifested the opposite trend (*p* < 0.05), implying that the renal function indexes are altered apparently in the case of renal injury, predicting the occurrence and development of the disease.

**Table 2.** Changes in the content of Cr, BUN, etc

Group	Cr(umol/L)	BUN(mmol/L)
Sham group Inhibitors group	20.12 ± 2.01 90.38 ± 2.07	7.19 ± 1.04 30.12 ± 3.51
Mimics group	35.87 ± 5.11 ^a^	13.04 ± 1.32 ^a^

Note: The content of Cr and BUN in the Mimics group decreased significantly, while the content in the Inhibitors group was opposite (P < 0.05) *P < 0.05 VS Sham, #P < 0.05 VS Inhibitors.

### 2.3 HE staining

The HE staining results are shown in Figure 2. There was glomerular injury, glomerular hypertrophy, renal proximal tubular damage, obviously thickened glomerular basement membrane, cystic dilation of renal tubule, apparent vacuolization of renal tubular epithelial cells, renal tubular hyalinization and renal cell injury in Inhibitors group (Figure 2a). In Mimics group, the renal glomerulus and renal tubule had normal morphology, and the renal tissue structure, histological structure and glomerular nodules were normal, without pathological changes observed (Figure 2b).

**Figure 2.** HE staining, glomerular damage, glomerular hypertrophy and proximal tubule damage in the Inhibitors group. Then the kidney cells were damaged (Figure A 20X). The glomeruli and tubules in the Mimics group were in normal shape, and no pathological changes were observed (Figure B 20X).

The article "Protective effect of MiR-146 on renal injury following cardiopulmonary bypass in rats through mediating NF-κB signaling pathway" was retracted in 2024. Reasons: original data or images not available; unreliable results or conclusions; concerns about the data; concerns about the results or conclusions.

### 2.4 Detection results of cytokines in each group

The levels of serum inflammatory factors such as TNF-α, IL-6 and IL-1 in the case of renal injury were determined (Table 3). It was shown that the levels of the three factors were elevated remarkably in Inhibitors group compared with those in the other two groups, while they declined obviously in Mimics group (*p* < 0.05), manifesting that overexpressed miR-146 cab inhibits the production of inflammatory factors.

**Table 3.** Test results of cytokines

Group	IL-1(mg/l)	TNF-α(fmol/ml)	IL-6(mg/l)
Sham	70.38 ± 4.45	38.10 ± 5.33	75.70 ± 3.20
Inhibitors	136.43 ± 5.07 ^a^	80.18 ± 4.07 ^a^	155.35 ± 5.55 ^a^
Mimics	80.93 ± 2.08 ^b^	44.79 ± 5.04 ^b^	89.38 ± 3.12 ^b^

Note: IL-6, TNF-α, IL-1 increased significantly in the Inhibitors group, and decreased significantly in the Mimics group (P < 0.05). (P < 0.05), a means P < 0.05 VS Sham; b means P < 0.05 VS Inhibitors.

### 2.5 Detection results of SOD and MDA in renal tissues

According to the results of SOD and MDA (Table 4), the content of MDA was raised in Inhibitors group (*p* < 0.05) and lowered in Mimics group (*p* < 0.05), but the opposite trends of SOD content were detected (*p* < 0.05).

**Table 4.** Kidney tissue SOD and MDA test results

Group	SOD (u/mg)	MDA (mmol/g)
Sham	50.5 ± 4.0	5.5 ± 1.4
Inhibitors	20.2 ± 3.4 ^a^	13.4 ± 2.5 ^a^
Mimics	40.5 ± 3.8 ^b^	7.8 ± 1.7 ^b^

Note: Oxidation and antioxidant index: MDA content increased in the Inhibitors group (P < 0.05), and decreased in the Mimics group (P < 0.05).

### 2.6 Expressions of related genes and pathway molecules in renal injury

As shown in Figure 3, the detection results of the gene expression indicated that the expression levels of vital gene ICAM-1, inflammatory gene TNF-α and pathway-related gene NF-κB during the progression of renal injury were reduced notably (*p* < 0.05), but the expression level of anti-oxidant gene SOD was raised markedly (*p* < 0.05) in Mimics group. However, the opposite expression levels were detected in the Inhibitors group, illustrating that reporter genes play pivotal roles in the process of renal injury, and pathway-related genes may be activated in the pathogenesis, thus indicating the further development of renal injury.

**Figure 3.** Gene expression results During the development of renal injury, the expression of important genes ICAM-1, inflammation gene TNF-α and pathway gene NF-KB were significantly reduced in the Mimics group (P < 0.05). Oxidative antioxidant gene SOD increased significantly (P < 0.05), a means P < 0.05 VS Sham; b means P < 0.05 VS Inhibitors.

### 2.7 TUNEL staining results

As shown in Figure 4, there were no obvious positive cells in the Sham group, the apoptosis rate in the Inhibitors group was significantly higher than that in the Sham group (P < 0.05), and the apoptosis rate in the Mimics group was significantly reduced (P < 0.05).

The article "Protective effect of MiR-146 on renal injury following cardiopulmonary bypass in rats through mediating NF-κB signaling pathway" was retracted in 2024. Reasons: original data or images not available; unreliable results or conclusions; concerns about the data; concerns about the results or conclusions.

**Figure 4.** TUNEL staining. No obvious positive cells were seen in the Sham group. The apoptosis rate in the Inhibitors group was significantly higher than that in the Sham group (P < 0.05), and the apoptosis rate in the Mimics group was significantly reduced (P < 0.05).

### 2.8 Expression of pathway-related protein

To further determine the impact of renal injury on the NF-κB signaling pathway, the protein expression levels were detected, and it was manifested that the expression level of the pathway protein NF-κB declined obviously in the Mimics group (*p* < 0.05), suggesting that the overexpression of miR-146 can accelerate the recovery of renal injury (Figure 5).

**Figure 5.** The expression level of the pathway protein NF-κB declines obviously in Mimics group (*p* < 0.05). ^a^*p*<0.05 vs. Sham group, ^b^*p*<0.05 vs. Inhibitors group. (a) Western blot result. (b) Quantification analysis of Western blot result.

Figure 5 the expression of pathway protein NF-KB in the Mimics group was significantly reduced (P < 0.05). a means P < 0.05 VS Sham; b means P < 0.05 VS Inhibitors.

### 2.9 Experimental analysis of dual luciferase

Dual luciferase experiments show that MIR-146 Mimics can significantly inhibit the luciferase activity of wild-type NF-KB plasmid, that is, inhibit the transcription activity of NF-KB, but has no obvious inhibitory effect on the luciferase activity of mutant NF-KB plasmid. This proves that MIR-146 can bind to the 3ʹUTR region of NF-KB, and NF-KB is the target gene of MIR-146, as shown in Table 5.

**Table 5.** Experimental analysis of dual luciferase

Group		Luciferase activity
Inhibitors group	NF-KB-WT	0.99 ± 0.15
	NF-KB-MUT	1.02 ± 0.12
Mimics group	NF-KB-WT	0.51 ± 0.16
	NF-KB-MUT	1.01 ± 0.18

## 3 Discussion

AKI will trigger various secondary reactive diseases in the severe stage, and early accurate diagnosis is the key to successful treatment and improvement of prognosis. MiR-146 can participate in the regulation of the CPB-associated renal injury, whose major role is to negatively regulate the immuno-inflammatory responses and exert a crucial effect in cell proliferation. Nevertheless, there is still limited evidence for the role and regulatory mechanism of miR-146 in AKI. Moreover, the function and specific mechanism of miR-146 in AKI have not been clarified yet. In the present study, the rat model of CPB was established, and miR-146 was silenced or overexpressed to further observe whether miR-146 plays a role in the CPB-associated renal injury, hoping to seek for potential therapeutic methods. Such a model has a similar physiological process of AKI to that in human, so it can be used as a favorable research object. The gene expression levels were detected to observe the transfection efficiency of miR-146 in each group of rats, and the results indicated that the expression level of miR-146 was elevated notably in Mimics group and lowered markedly in Inhibitors group, suggesting that the transfection efficiency was prominent, and related verification tests could be further conducted. In addition, the important biochemical indexes (Cr and BUN) in the serum have vital functions in nephropathy. The results in this study showed that Mimics group exhibited evidently decreased content of Cr and BUN, while Inhibitors group manifested the opposite trend, implying that the renal function indexes are changed prominently when renal injury occurs, predicting the occurrence and development of the disease. Those results are consistent with those in previous studies [18].

The article "Protective effect of MiR-146 on renal injury following cardiopulmonary bypass in rats through mediating NF-κB signaling pathway" was retracted in 2024. Reasons: original data or images not available; unreliable results or conclusions; concerns about the data; concerns about the results or conclusions.

The AKI associated with extracorporeal circulatory surgery is complex, including multiple synergistic damage pathways, including ischemia-reperfusion injury, exogenous and endogenous toxins, inflammation, oxidative stress, and hemodynamic factors [19]. Apoptosis plays an important role in the occurrence and development of AKI. Previous studies have found that during the occurrence of AKI, cell apoptosis is related to inflammation, and inflammation produces a large amount of inflammatory factors such as TNF-α, IL-6, IL-1, etc. These inflammatory factors can be used as the initiating factors of apoptosis and activate the apoptosis pathway, thereby mediating the death of renal tubular cells [20]. In this experiment, the levels of serum inflammatory factors such as TNF-α, IL-6 and IL-1 in the case of renal injury were determined. It was discovered that the levels of the three factors were elevated remarkably in Inhibitors group compared with those in the other two groups, while they declined obviously in Mimics group, manifesting that overexpressed miR-146 cab inhibit the production of inflammatory factors. Under the action of free unstable iron, the I/R injury induced by the CPB-associated oxidative stress may be aggravated furthermore. The non-physiological surface and shear stress of the CPB circuit can cause mechanical damage to the erythrocytes and release the free hemoglobins into the circulation [21]. With the presence of oxidants, the free iron can be released from heme that contains redox-active iron capable of stimulating lipid peroxidation, catalyzing the formation of hydroxyl radicals and thus damaging the tissues [22]. The free unstable iron can arouse a variety of changes in the renal tubular epithelial functions, including impaired proliferation and induced free radical injury. Such an association is probably related to hemolysis and generation of free hemoglobins and free toxic iron in the blood vessels [23]. The detection of oxidative stress in this study revealed that the content of MDA was increased in Inhibitors group but decreased in Mimics group, and the opposite trends of SOD were detected, which are in line with the findings in the above studies. Pigment nephropathy results from hemoglobinuria and myoglobinuria. The increased hemoglobins in the plasma during CPB are related to postoperative renal tubular damage in the early stage and independently associated with subsequent AKI [24]. The HE staining results showed that Inhibitors group had glomerular injury, glomerular hypertrophy, renal proximal tubular damage, obviously thickened glomerular basement membrane, cystic dilation of renal tubule, apparent vacuolization of renal tubular epithelial cells, renal tubular hyalinization and renal cell injury. In Mimics group, however, the renal glomerulus and renal tubule were normal in morphology, with normal renal tissue structure, histological structure and glomerular nodules and without pathological changes observed. TUNEL staining revealed that there were no obvious positive cells in the Sham group. The apoptosis rate in the Inhibitors group was significantly higher than that in the Sham group. The apoptosis rate in the Mimics group was significantly reduced, which are in line with the aforementioned results.

The article "Protective effect of MiR-146 on renal injury following cardiopulmonary bypass in rats through mediating NF-κB signaling pathway" was retracted in 2024. Reasons: original data or images not available; unreliable results or conclusions; concerns about the data; concerns about the results or conclusions.

The dysregulated NF-κB signal transduction mechanism is the potential pathogeny of numerous diseases [25]. Hence, it is essential to understand the relationship between NF-κB and downstream signaling molecules. As a switch or inductor, NF-κB can produce the inflammatory responses to various stimulations and initiate the inflammatory genes [26]. A study has demonstrated that ICAM-1 plays an important role in renal injury and can act as a vital detection index, whose expression level will be elevated in the case of renal injury [27,28]. In the present study, the detection results of the gene expression indicated that the expression levels of vital gene ICAM-1, inflammatory gene TNF-α and pathway-related gene NF-κB during the progression of renal injury declined notably, but the expression level of anti-oxidant gene SOD rose markedly in Mimics group. However, Inhibitors group displayed the opposite expression levels, illustrating that reporter genes exert pivotal effects in the process of renal injury, and pathway-related genes may be activated during the onset of the disease, thus indicating the further development of renal injury. In order to further confirm the impacts on the key molecules and the NF-κB signaling pathway in the process of renal injury, the expression levels important proteins were measured, and it was manifested that the expression level of the pathway protein NF-κB declined obviously in Mimics group during the progression of renal injury, suggesting that the overexpression of miR-146 can accelerate the recovery of renal injury. It was proven in this study that up-regulating the expression of miR-146 can inhibit the secretion of inflammatory factors, resist oxidative stress and repress the expression of the NF-κB signaling pathway, thereby promoting the recovery of renal injury after CPB. Nonetheless, there were also some deficiencies in this study. For example, only in-vivo experiments instead of more cell culture experiments in vitro were performed to mutually verify the impacts of miR-146 on the repair of renal injury and the NF-κB signaling pathway. This study proved that up-regulation of MIR-146 expression can inhibit the secretion of inflammatory factors, fight oxidative stress, inhibit the expression of NF-KB pathway, and promote the recovery of renal injury after PCB. Dual luciferase experiments show that MIR-146 can bind to the 3ʹUTR region of NF-KB, and NF-KB is the target gene of MIR-146. But our research also has certain shortcomings. For example, no more in vitro cell culture experiments have mutually confirmed the effect of MIR-146 on the repair of kidney injury.

The article "Protective effect of MiR-146 on renal injury following cardiopulmonary bypass in rats through mediating NF-κB signaling pathway" was retracted in 2024. Reasons: original data or images not available; unreliable results or conclusions; concerns about the data; concerns about the results or conclusions.

## 4. Conclusion

Cellular oxidative stress occurs when kidney injury occurs in vitro circulation, which induces a series of pathological changes such as apoptosis, increased inflammation, renal dysfunction, and activation of inflammatory pathways. Up-regulation of MIR-146 can inhibit the occurrence of diseases by inhibiting the NF-KB signaling pathway. The progress of this study provides a theoretical basis for the prevention and treatment of renal damage in vitro.

## Data Availability

The datasets used and/or analyzed during the current study are available from the corresponding author on reasonable request.
